# Effects and Action Mechanism of Huoxue Tongluo Formula on the Formation of Neutrophil Extracellular Traps

**DOI:** 10.1155/2022/1240967

**Published:** 2022-08-18

**Authors:** Xiaoli Zhou, Weixiang Liao, Wei Peng, Tingting Xie, Qianlu Yin, Yuhang Zheng

**Affiliations:** ^1^Department of Peripheral Vascular (Wound Repair), Chongqing Hospital of Traditional Chinese Medicine, Chongqing 400021, China; ^2^Graduate School, Guizhou University of Traditional Chinese Medicine, Guiyang 550002, China

## Abstract

Excessive infiltration and uncontrolled activation of neutrophil extracellular traps (NETs) are likely to destroy normal tissue architecture and cause uncontrolled inflammation. The present research attempted to screen potential signaling pathways of Huoxue Tongluo Formula (HXTLF) affecting the formation of NETs using network pharmacology technique. Active chemical components of HXTLF and therapeutic targets related to vasculitis were screened, and a chemical components-targets network diagram of HXTLF was constructed by Cytoscape. Finally, the inhibitory effect and mechanism of HXTLF on the formation of NETs were explored in vitro using LPS-induced NETs. Immunofluorescence and Western blot were conducted to determine the protein fluorescence intensity and relative expression. The experimental results illustrated that HXTLF mediated the expression levels of H3Cit and myeloperoxidase (MPO) protein in neutrophils activated by LPS, inhibited NETs formation, and reduced the concentration of interleukin- (IL-) 1*β*, a proinflammatory factor in cells. Additionally, we activated and inhibited the AKT1 signaling pathway using the corresponding activator and inhibitor to explore the regulatory mechanism of HXTLF on AKT1 and other molecules in the treatment of vasculitis. The results demonstrated that HXTLF could inhibit the phosphorylation of AKT1, IKK, and NF-*κ*B proteins, inhibit NETs formation, and reduce IL-1*β* concentration, indicating that AKT1 exerts a vital role in the treatment of vasculitis after HXTLF administration. The current study initially revealed the pharmacological mechanism of HXTLF for vasculitis management using network pharmacology techniques and tests in vitro, which is expected to provide important theoretical basis for elucidating the molecular mechanism of HXTLF and promoting its clinical application.

## 1. Introduction

Neutrophils produce innate immune functions mainly through phagocytosis, degranulation of phagosomes, and neutrophil extracellular traps (NETs). NETs are reticular complexes including free DNA, histones, and neutrophil granule proteins, which can trap invading pathogens and degrade pathogens through NETs-associated proteolytic enzymes [1]. As the immune defense function of neutrophils remains after death, these cells have become a research hotspot by researchers and scholars since being discovered by Brinkmann et al. in 2004 [2]. After 18 years of research, NETs are commonly found in inflammatory diseases, infectious and noninfectious diseases, autoimmune diseases, cancer, and other diseases [3]. NETs formation is found activated by LPS in some studies, which promotes the secretion of inflammasomes IL-18, IL-1*β*, and NOD-like receptor thermal protein domain associated protein 3 (NLRP 3). In addition to promoting inflammatory responses, these cytokines can further induce the formation of NETs [4]. Meanwhile, NETs also interact with other adaptive immune cells, namely, B cells, T cells, as well as antigen-presenting cells. Palanichamy et al. have pointed out that interferon- (IFN-) *ɑ* produced by bone marrow neutrophils can inhibit the development of B cells in early systemic lupus erythematosus [5]. The research of Sawalha has reported that neutrophils from patients with systemic lupus erythematosus activate dendritic cells (DCs) and release their own antigens in NETs through toll-like receptor 9 (TLR 9) [6]. As NETs may be central regulators of inflammatory responses, they are expected to be novel biomarkers and therapeutic targets for inflammatory diseases.

Huoxue Tongluo Formula (HXTLF) is written in “Zhu Renkang Clinical Experience Collection.” The main compositions of the formula include Danggui (*Angelicae sinensis Radix*), Honghua (*Carthamus tinctorius* L.), Taoren (*Persicae Semen*), Chishao (*Paeoniae radix Rubra*), Qiancao (*Rubia cordifolia* L.), Niuxi (*Achyranthes bidentata Blume*), Zelan (*Eupatorium* L.), Qingpi (*Citri reticulatae Pericarpium viride*), and Xiangfu (*Cyperus rotundus* L.), 9 g for each composition. HXTLF is mainly introduced to treat diseases of qi stagnation and blood stasis, erythema nodosum, erythema induration, and sarcoidosis of the lower extremities. The active ingredients of this formula have also achieved satisfactory effects on immune regulation, reversal of chronic inflammation, and inhibition of abnormal cell proliferation [7–10]. However, the interrelationship between HXTLF and NETs remains to be fully elucidated.

Data mining of HXTLF components and target prediction are the basic work of applying network pharmacology technique. According to the Traditional Chinese Medicine Systems Pharmacology Database and Analysis Platform, chemical database, disease database, target database, genome database, and functional protein connection network database, the effective components of HXTLF were screened out, potential functional targets were predicted, and the network diagram of “drug-target-disease” was plotted. Meanwhile, the pharmacological mechanism of “multicomponents, multitargets, and multipathways” was elucidated, which has become an indispensable aspect in the research of traditional Chinese medicine network pharmacology. This study's aim was to investigate the effect and mechanism of HXTLF on the formation of NETs using a network pharmacology technique.

## 2. Materials and Methods

### 2.1. Network Pharmacology

Based on the principles of network pharmacology, major chemical components of HXTLF were firstly obtained including *Carthamus tinctorius* L., *Achyranthes bidentata Blume*, *Cyperus rotundus* L., *Persicae semen*, *Rubia cordifolia* L., *Paeoniae Radix Rubra*, *Citri reticulatae Pericarpium viride*, the last part of *Angelicae Sinensis Radix*, and *Eupatorium* L., from the TCMSP website (https://old.tcmsp-e.com/tcmsp.php), and the corresponding action targets were predicted. The selection of the main active ingredients was oral bioavailability (OB) ≥ 30% and drug likeness (DL) ≥ 0.18 [11]. All targets of the active ingredients are downloaded from Swiss TargetPrediction website [12]. Meanwhile, disease targets associated with human immune small vasculitis were exported from genetic disease database; a protein-protein interaction (PPI) network was plotted via String, an online platform. Subsequently, a drug-component-target-disease network diagram was also constructed via Cytoscape 3.6.0 software. Furthermore, GO and KEGG pathway enrichment were analyzed using ClueGO, a plugin of Cytoscape on the overlapped genes, and finally the enrichment results were presented for analysis.

### 2.2. Preparation of Serum Containing HXTLF

The serum containing HXTLF was prepared by the establishment of a model of SD rats. Six SPF-grade SD rats aged 8 weeks were from Chongqing Ensiweier Biotechnology Co., Ltd. They were divided into blank and HXTLF groups, three of each, which were intragastrically administered with distilled water and HXTLF at 10 times of the clinical dose and lasted for consecutive 7 days [13]. The abdominal aortic blood samples were obtained, serum was separated, and complement was inactivated.

### 2.3. Neutrophil Induction and Grouping

Neutrophils are collected by density gradient centrifugation [14]. Briefly, 2 mL EDTA anticoagulant was used, and red blood cell lysate (R1010, Solarbio) was added at 1 : 3 under a sterile condition, mixed thoroughly and let stand for 15 min. Following centrifugation at 1 000 r/min for 5 min, the supernatant was abandoned. Lysis of red blood cells was repeated once. The white blood cells at the bottom of the tube were reserved, supplemented with 2 mL of PBS containing 1% BSA, mixed well, and transferred to the liquid surface of a 4 mL 60% Percoll (P8370, Solarbio) tube, centrifuged at 2 000 r/min for 20 min, and neutrophils were deposited at the bottom of the tube. The neutrophils were collected after two cycles of washing using PBS containing 1% BSA and then diluted to 200 *μ*L for subsequent use. The neutrophils were cultured in DMEM medium (L110 KJ, Basal Media) containing 1% penicillin-streptomycin (C0009, Beyotime) and 10% FBS (AC03L055, Life-iLab) at 37°C in a 5% CO_2_ incubator.

During the experiment, neutrophils were divided into 5 groups: control, model, LPS + low (2.5%), medium (5%), and high (10%) HXTLF dose groups. The model group was LPS-induced at 100 ng/ml and lasted 4 h to stimulate NETs formation, the control group was added with serum of the blank group, and the HXTLF groups were treated with LPS + HXTLF at several concentrations. The cells and supernatant were collected after 4 h for tests.

### 2.4. Immunofluorescence

Followed by a cycle of washing using distilled water, sample sections were immersed in PBS for 5 min, positioned with 4% paraformaldehyde for 15 min, and cleaned with PBS for three times, each time for 3 min. After the addition of 0.5% TritonX-100 (ST795, Beyotime), the sections were drilled for 10 min at room temperature, immersed in PBS 3 min for three repeats, provided with normal goat serum (C0265, Beyotime) dropwise, and blocked 60 min at room temperature.

The blocking solution removal was conducted using a piece of absorbent paper and the cells were added with sufficient diluted primary antibody (Abcam, Shanghai) by drips, kept in a wet chamber for incubation at 4°C overnight. The slides were taken out with the wet box, kept at room temperature for 30 min, and soaked in PBS three times, each time 3 min. After the removal of excessive solution with absorbent paper, fluorescent secondary antibodies were supplemented after being diluted to an appropriate proportion and placed in the wet box again for incubation at 37°C for 60 min. Following immersion in PBS for three times, DAPI was supplied by drips and incubated for 15 min in the dark. Cell nucleus staining was performed, and then followed by four cycles of PBS washing to remove excess DAPI, each time lasting for 5 min. The slides were subsequently sealed with antifluorescence quencher dropwise, and image acquisition was performed using a fluorescence microscope (OLYMPUS, Japan).

### 2.5. NETs Cell Free DNA Detection

The detection of NETs in peripheral blood was determined by circulating free DNA (cfDNA) fluorescent staining. Experiments were performed according to the PicoGreen dsDNA quantitative detection kit (Solarbio, China). Briefly, 1 mg/mL calf thymidine DNA dry powder (Sigma) standard working solution and PicoGreen dye working solution were first prepared. 1 mg/mL calf thymine DNA dry powder standard working solution was double diluted, and the fluorescence value of the sample was detected by a fluorometer. The excitation and emission wavelength were measured at 488 nm and 520 nm, respectively. The working curve of the standard product was drawn, and the sample was measured; NETs concentration was determined.

### 2.6. ELISA

The collected complete blood samples were kept at room temperature for 2 hours, centrifuged at 1000 g for 20 min for serum collection, and stored at −80°C. The serum IL-1*β* concentration was detected by using Rat IL-1*β* ELISA KIT as per the manufacturer's instructions (RX106152H, Ruixin BioTech).

### 2.7. Western Blot

By adding RIPA cell lysate containing protease inhibitor, total protein was extracted, vortexed evenly, cultured on ice for 20 min, and the protein concentration was determined by a BCA method. After an addition of 5× loading buffer and mixing well, the protein was boiled at 100°C for 5 min for denaturation and electrophoresis separation was performed at 90V. Following the electrophoresis, the protein was transferred onto a PDVF membrane using constant current of 300 mA. The PDVF film blocking was carried out at room temperature for 2 h using TBST blocking solution containing 5% skimmed milk. After the blocking agent was removed, primary antibodies were diluted and added for culture overnight on a 4°C shaker. After three cycles of TBST rinsing, each time for 8 min, secondary antibodies (AS014, ABclonal) were provided, incubated at room temperature for 1.5 h, and followed by a cycle of TBST washing. Ultimately, ECL chemiluminescence detection kit with a Tanon-4500 chemiluminescence system are used for development. The primary antibodies included AKT (A11016, ABclonal); p-AKT (AP0637, ABclonal); IKK (A2062, ABclonal); p-IKK (AP0505, ABclonal); NF-*κ*B (10745-1-AP, ABclonal); p–NF–*κ*B (3033T, ABclonal); and *β*-Actin (AC026, ABclonal).

### 2.8. Statistical Analysis

Three independent experiments were carried out. The obtained data were analyzed using GraphPad Prism 8.0.1 and expressed as mean ± standard deviation (SD). Groupwise comparisons of one-way ANOVA analysis were performed using Tukey's tests (*n* = 3). *P* < 0.05 was considered significant difference.

## 3. Results

### 3.1. GO and KEGG Analysis of Small Vasculitis Treatment Using HXTLF

HXTLF is effective in rheumatoid arthritis management clinically [15]. To explore whether HXTLF acts on small vasculitis, the active components were identified, and relevant drug targets were predicted. The active components (*Carthamus tinctorius* L., *Achyranthes bidentata Blume*, *Cyperus rotundus* L., *Persicae Semen*, *Rubia cordifolia* L., *Paeoniae Radix Rubra*, *Citri Reticulatae Pericarpium Viride*, the last part of *Angelicae Sinensis Radix*, and *Eupatorium* L.) of HXTLF were retrieved from TCMSP and corresponding targets were predicted from the Swiss TargetPrediction website. A total of 684 targets in HXTLF were obtained. There were 191 targets for small vasculitis collected in the genetic disease database, of which 43 targets overlapped with the active components of HXTLF (Figure 1(a)). PPI network diagram was exported from online platform String (Figure 1(b)). Subsequently, the forty-three overlapping targets of HXTLF and the disease were analyzed to clarify their functions and possible roles in signaling pathways using GO and KEGG enrichment analysis and the enrichment results were presented. The GO findings suggested that more significant GO terms included positive regulation of cell activation, T-cell activation, regulation of cell-cell adhesion, and positive regulation of cell adhesion in the biological process. The effects on phosphatase binding, cytokine receptor binding, and protein serine/threonine kinase activity were more pronounced in molecular function (Figure 1(c)). KEGG pathway enrichment revealed that the forty-three overlapping targets of HXTLF against vasculitis were annotated to PI3K-Akt signaling pathway and HIF-1 signaling pathway (Figure 1(d)).

### 3.2. Hub Gene Network Diagram

To present a more vivid profile of the interrelationship of drugs, components, targets, and the disease and to predict possible action targets of the drugs, we obtained twenty hub genes from the PPI network analysis and constructed a network diagram of drug-active components-targets-disease through Cytoscape, as shown in Figure 2. Based on PPI analysis, the overlapped genes with higher degrees in the hub gene network included MAPK1, MAPK3, VEGFA, TNF, and AKT1, implying that they were involved in the process of HXTLF treatment against vasculitis.

### 3.3. HXTLF Inhibits the Formation of NETs

After the collection of rats' peripheral blood samples, density gradient centrifugation was performed to obtain neutrophils, which were cultured subsequently. The rats were simultaneously administered 10 times the clinical dose of HXTLF by gavage for 7 consecutive days to obtain the HXTLF-contained serum of the rats. Through an addition of the same dose as double distilled water to the blank group, serum was collected. The experiments had classified neutrophils into five groups. The rats in the blank group were treated with serum for blank group to interfere with cell growth, rats in the model group were administrated with LPS to induce the formation of NETs, and the HXTLF groups were given with different concentrations (2.5%, 5%, and 10%) of rat serum containing HXTLF, to clarify the effect on the formation of NETs. Cellular H3Cit and myeloperoxidase (MPO) were detected using immunofluorescence, and the mean fluorescence intensity was calculated (Figure 3(a)), indicating that the fluorescence intensity of H3Cit and MPO was elevated substantially in the model group versus control group. Being processed with serum containing different concentrations of HXTLF, the fluorescence of H3Cit and MPO in the HXTLF group decreased in a dose-dependent manner. Meanwhile, PicoGreen dsDNA quantitative detection kit was used to determine the content of free DNA in the cell supernatant. The release of NETs in the model group increased largely versus control and serum containing HXTLF could inhibit the release of NETs in a dose-dependent fashion. As the concentration of HXTLF increased, its inhibitory effect was more satisfactory (Figure 3(b)). The above results suggested that serum containing HXTLF could inhibit the formation of NETs, and the best curative effect was achieved in the 10% HXTLF group. Furthermore, the concentration of proinflammatory factor IL-1*β* in the supernatant was determined, which was markedly elevated in the model group, whereas it decreased after HXTLF treatment, and the difference was significant as compared to control (Figure 3(c)).

### 3.4. HXTLF Inhibits the Formation of NETs by Regulating AKT

The previous experiments investigated the effect of HXTLF on the formation of NETs, and the results revealed that HXTLF could inhibit the formation of NETs, and the best curative effect was achieved in the 10% HXTLF group. We predicted potential targets of HXTLF for vasculitis management using network pharmacology. We attempted to elucidate how HXTLF affected the formation of NETs and the relevant molecular mechanism, AKT activator (SC79), and inhibitor (MK-2206 2HCl) were used to interfere with the growth of neutrophils during the experiments. The cells were divided into six groups as per the addition of AKT activator and inhibitor or not as following: model group (LPS + blank serum), HXTLF group (LPS+10% HXTLF), model + activator group (SC79 + LPS + blank serum), HXTLF + activator group (SC79 + LPS + +10% HXTLF), model + inhibitor group (MK-2206 2HCl + LPS + blank serum), and HXTLF + inhibitor group (MK-2206 2HCl + LPS + 10% HXTLF). The expression of AKT1, IKK, and NF-*κ*B and the corresponding protein phosphorylation were determined using Western blotting, as presented in Figure 4(a). The expression of p-AKT1, p-IKK and p-NF-*κ*B proteins in the model + activator group was largely elevated versus the model, whereas that of the model + inhibitor group was markedly decreased. AKT activator and inhibitor could greatly upregulate and downregulate p-IKK and p-NF-*κ*B levels in neutrophils, respectively. Additionally, the HXTLF group could significantly reduce p-AKT1, p-IKK, and p-NF-*κ*B protein levels in neutrophils as compared to model. After AKT1 activator pretreatment, p-AKT1, p-IKK, and p-NF-*κ*B levels in cells were markedly higher than model but lower than model + activator group. After inhibitor pretreatment, the expression of the described three proteins in the HXTLF + inhibitor group was substantially lower versus model. The same results were obtained as compared to the HXTLF group.

Additionally, immunofluorescence was performed to determine H3Cit and MPO protein fluorescence in cells of each group, and the mean fluorescence intensity was calculated. As shown in Figure 4(b), the fluorescence intensity of H3Cit and MPO proteins in the model + activator group was significantly increased, but largely declined in model + inhibitor group versus model group, implying that AKT might play a role in regulating NETs formation. Conversely, the fluorescence intensity of H3Cit and MPO protein in neutrophils in the HXTLF-treated group was substantially decreased as compared to model. After AKT1 activator pretreatment, the fluorescence intensity of H3Cit and MPO proteins in cells was significantly increased versus model whereas decreased versus model + activator. After inhibitor pretreatment, the fluorescence intensities of H3Cit and MPO proteins in the HXTLF + inhibitor group were markedly decreased as compared to model and the fluorescence intensity of H3Cit and MPO proteins also decreased when compared with the HXTLF group.

The content of free DNA of NETs and the proinflammatory factor IL-1*β* in cells were evaluated. The trend in each group was in agreement with the previously described findings of Western blotting and immunofluorescence. HXTLF could hinder the formation of NETs; activation and inhibition of AKT1 pathway could affect the formation of NETs and the efficacy of HXTLF in inhibiting the formation of NETs (Figures 4(c)–4(d)).

## 4. Discussion

Neutrophils have innate immune function, and the released NETs can capture and kill bacteria [16]. The basic components of NETs, PR3, and MPO have immunogenicity and are involved in the onset of antineutrophil cytoplasmic antibody associated vasculitis (AAV) [17]. AAV belongs to systemic immune disorder in the presence of inflammation as well as fibrinoid necrosis in small blood vessel walls, namely, microscopic polyangiitis, granulomatosis with polyangiitis, and eosinophilic granulomatosis with polyangiitis [18, 19]. This disease progress is rapid and its prognosis is very dangerous. In particular, antineutrophil cytoplasmic antibody can combine with MPO on the surface of neutrophils, which are activated by proinflammatory factors, and further promote neutrophil activation, release more NETs, and aggravate AAV forming a vicious circle.

Excessive infiltration and uncontrolled activation of NETs might result in the destruction of normal tissue structure and uncontrolled inflammation, thus leading to several acute inflammatory responses [20]. Studies have shown that the formation of NETs in diffuse large B-cell lymphoma directly upregulates toll-like receptor 9 pathway, thereby activating the STAT3, NF-*κ*B, and p38 pathways to facilitate tumor progression, which suggests that NETs might be a prognostic marker for tumors [21]. Some researchers have pointed out the role of NETs in the pathogenesis of autoimmune diseases. Except for AAV, patients with systemic lupus erythematosus also have excessive NETs formation [22]. By providing scaffolds and stimulating the adhesion and aggregation of platelets and erythrocytes, vascular compartment NETs can promote thrombus formation, and all the major components are characterized by their procoagulant properties that can mediate thrombus formation [23, 24]. It can be seen that the inhibition of NETs formation exerts a positive effect on autoimmune diseases and inflammatory processes. Meanwhile, the mechanism exploration of NETs formation is essential to inhibit the formation, thereby alleviating the disease process of vasculitis.

The main active components of HXTLF and the disease targets of vasculitis were screened, and a diagram of drug-components-targets-disease of HXTLF was established using software Cytoscape 3.7.2, and hub genes were analyzed based on the PPI network diagram. Meanwhile, the common targets and relevant signal pathways involved in both networks were analyzed through GO function and KEGG pathway enrichment, suggesting that the effects of HXTLF on positive regulation of cell activation, regulation of cell-cell adhesion, positive regulation of cell adhesion, and T cell activation were more significant during the GO biological process. The effects on protein serine/threonine kinase activity, cytokine receptor binding, and phosphatase binding were also significant in molecular function. KEGG pathway analysis revealed that HXTLF was associated with HIF-1 and PI3K-Akt signaling pathways for vasculitis management. The PI3K/Akt signaling pathway can mediate various cell functions, namely, metabolism, growth, proliferation, and survival. Its abnormal activation can trigger the occurrence and development of various tumors, leading to insulin resistance, and affecting skeletal muscle, adipose tissue, liver, skeletal muscle, adipose tissue, and the brain. Meanwhile, it also relates to metabolic diseases, namely, type 2 diabetes and obesity [25, 26]. Recent research has reported that PI3K/Akt inhibitors can inhibit the formation of NETs in polymorphonuclear neutrophils stimulated by PMA and SLE serum, suggesting that PI3K/Akt exerts a role in the formation of NETs in SLE patients.

We used LPS to induce the formation of neutrophil NETs in vitro to elucidate the inhibitory effect and mechanism of HXTLF associated with its formation. Subsequent experimental results verified the effect of HXTLF on inhibiting the formation of NETs in cells, reducing the fluorescence intensity of intracellular H3Cit and MPO proteins, decreasing the content of free DNAs as well as the concentration of IL-1*β*, the proinflammatory factor in cells. Furthermore, we supplemented AKT1 activator (SC79) and inhibitor (MK-2206 2HCl) to interfere with the neutrophil growth, respectively, and discussed the relevant regulatory mechanism of HXTLF on vasculitis treatment. It indicated that HXTLF could inhibit the phosphorylation of cellular AKT1, IKK, and NF-*κ*B proteins, hamper the formation of NETs, and reduce cell-induced IL-1*β* generation. The IKK kinase complex is essential for NF-*κ*B cascade. I*κ*B molecules usually interact with NF-*κ*B and remain inactive in the cytoplasm. After being stimulated by inflammatory cytokines, bacterial or viral products, I*κ*B is phosphorylated by IKK, thus allowing free NF-*κ*B to enter the nucleus and participate in immune and inflammatory responses [27]. In response to the invasion of microorganisms and the corresponding products, namely, LPS, immune cells secrete inflammatory mediator IL-1*β* to induce the expression of adhesion molecules on endothelial cells, thereby facilitating the recruitment of inflammatory cells to the inflammation sites [28]. As a typical inflammatory cytokine, IL-1*β* stimulates local and systemic inflammatory responses. Its antagonist prevents glomerulonephritis in a model of anti-MPO-induced rat, and the presence is important in the pathogenesis of vasculitis [29]. After MK-2206 2HCl pretreatment, HXTLF inhibited protein phosphorylation and NETs formation but increased the concentration of proinflammatory factor.

Though, this study validates the potential role of HXTLF in the treatment of vasculitis through network pharmacology techniques and in vitro tests. It helps to provide significant theory in elucidating the molecular mechanism of HXTLF on vasculitis and promoting HXTLF usage in clinical application as a new potential formula and further molecular mechanism within it. The limitations are inevitable; first, the specific substances or chemicals in serum containing HXTLF have not been explored and second, the potential role of AKT in vasculitis needs deeper investigation.

## 5. Conclusion

The present study preliminarily revealed the pharmacological mechanism of HXTLF in treating vasculitis using network pharmacology and in vitro experiments, implying that HXTLF might treat vasculitis by regulating AKT to inhibit the formation of NETs and induce IL-1*β* production in cells. It is regarded that AKT1 exerts an essential role in the treatment of vasculitis with HXTLF.

## Figures and Tables

**Figure 1:** Results of GO and KEGG enrichment analysis of the overlapped genes between HXTLF and small vasculitis. (a) Venn diagram. (b) PPI network diagram. (c) Bar charts of biological process, molecular function, and cellular component in GO analysis. GO terms are on the left, and abscissa represents gene count. (d) Circle diagram of KEGG pathway enrichment. The right outer layer indicates metabolic pathways and the left indicates genes. The left inner circle indicates *p* values for significance for the corresponding pathways.

**Figure 2:** Diagram of drug-active component-target-disease network between HXTLF and small vasculitis. (a) Hub gene network diagram; the color is changing from yellow to red; the darker represents the more nodes of the genes. (b) Diagram of drug-active component-target-disease network. The purple diamonds represent overlapped genes. The size of diamonds represents there are more connections between the genes and components. The V shape represents the main drugs of HXTLF. The regular hexagon represents the main active components of the drugs.

**Figure 3:** The influence of HXTLF on the formation of NETs. (a) Immunofluorescence microscopy of H3Cit and MPO, and bar charts on the right indicate mean fluorescence intensity. Magnification 400 ×. Scale bar is 50 *µ*m. (b) NETs cell free DNA detection. (c) Detection of secretion factor IL-1*β* in neutrophil supernatant. Significance was represented by asterisks: ^*∗*^*P* < 0.05; ^*∗∗*^*P* < 0.01 compared to control, *n* = 3.

**Figure 4:** Effect of HXTLF on the formation mechanism of NETs. (a) Western blot detection of the expression of AKT1, p-AKT1, IKK, p-IKK, NF-*κ*B, and p-NF-*κ*B in neutrophils (left). *β*-Actin was employed as an internal reference protein. Semiquantitative analysis was used for protein quantification and ImageJ was utilized to analyze the gray value of protein bands. The results were displayed in column diagram (right). (b) Immunofluorescence microscopy of H3Cit and MPO, and the right was mean fluorescence intensity calculated. Magnification 400 ×. Scale bars = 50 *µ*m. (c) NETs cell free DNA detection. (d) Detection of secretion factor IL-1*β* in neutrophil supernatant. Activator (pretreatment with SC79 in 8 *µ*g/ml for 30 min); Inhibitor (pretreatment with MK-2206 2HCl in 10 *µ*m/L for 30 min). DMSO was used as the activator and inhibitor control. The data were obtained from three independent experiments and expressed as mean ± SD. Asterisks indicated significance: ^*∗*^*P* < 0.05; ^*∗∗*^*P* < 0.01 compared to control, *n* = 3.

## Data Availability

The data used to support the findings of this study are included within the article.
